# Dictionary Learning-Based Ultrasound Image Combined with Gastroscope for Diagnosis of Helicobacter pylori-Caused Gastrointestinal Bleeding

This article has been retracted.

**DOI:** 10.1155/2021/6598631

**Published:** 2021-12-28

**Authors:** Yunyun Diao, Zhenzhou Zhang

**Affiliations:** Department of Digestion and Hematology, Sinopharm North Hospital, Baotou, 014030 Inner Mongolia, China

## Abstract

The study is aimed at evaluating the application value of ultrasound combined with gastroscopy in diagnosing gastrointestinal bleeding (GIB) caused by Helicobacter pylori (HP). An ultrasound combined with a gastroscopy diagnostic model based on improved *K*-means Singular Value Decomposition (N-KSVD) was proposed first. 86 patients with Peptic ulcer (PU) and GIB admitted to our Hospital were selected and defined as the test group, and 86 PU patients free of GIB during the same period were selected as the control group. The two groups were observed for clinical manifestations and HP detection results. The results showed that when the noise *ρ* was 10, 30, 50, and 70, the Peak Signal to Noise Ratio (PSNR) values of N-KSVD dictionary after denoising were 35.55, 30.47, 27.91, and 26.08, respectively, and the structure similarity index measure (SSIM) values were 0.91, 0.827, 0.763, and 0.709, respectively. Those were greater than those of DCT dictionary and Global dictionary and showed statistically significant differences versus the DCT dictionary (*P* < 0.05). In the test group, there were 60 HP-positives and 26 HP-negatives, and there was significant difference in the numbers of HP-positives and HP-negatives (*P* < 0.05), but no significant difference in gender and age (*P* > 0.05). Of the subjects with abdominal pain, HP-positives accounted for 59.02% and HP-negatives accounted for 37.67%, showing significant differences (*P* < 0.05). Finally, the size of the ulcer lesion in HP-positives and HP-negatives was compared. It was found that 71.57% of HP-positives had ulcers with a diameter of 0-1 cm, and 28.43% had ulcers with a diameter of ≥1 cm. Compared with HP-negatives, the difference was statistically significant (*P* < 0.05). In conclusion, N-KSVD-based ultrasound combined with gastroscopy demonstrated good denoising effects and was effective in the diagnosis of GIB caused by HP.

## 1. Introduction

Peptic ulcer (PU) is a common disease of the digestive system, and gastrointestinal bleeding (GIB) is the most common complication of PU, occurring in more than 25% of patients. Most patients have GIB before there is no abdominal pain [1, 2]. Relevant clinical studies have shown that chronic gastritis, PU, intestinal metaplasia, gastric cancer, and mucosa-associated lymphoid tissue are closely related to infection with helicobacter pylori (HP) [3, 4]. HP is a gram-negative microaerobion that can colonize gastric mucosa for a long time, and its pathogenic factors include virulence factors, cytokines, immunological factors, and genetic susceptibility of the body [5, 6]. HP has the fecal-oral access to the digestive tract, and secreted urea enzyme can decompose the urea in the stomach to produce large amounts of ammonia to adapt to acid environment in the stomach. Moreover, HP flagella can help it pass through the mucus to the mucosal surface of the stomach, causing the corresponding gastric mucosal inflammation which further leads to GIB [7–9]. In China, the high infection rate of HP is as high as 60%-80%. Therefore, the examination and diagnosis of HP are important [10, 11].

The current clinical methods to detecting HP infection include rapid urease test (RUT), staining microscopic examination of gastric mucosal tissue sections, ^13^C- or ^14^C-urea breath test (UBT), stool HP antigen detection, serum and secretion HP antibody detection, and polymerase chain reaction (PCR) [12–14]. With the development of ultrasonic diagnosis technology, some scholars have combined ultrasound and gastroscopy to detect the infection and bleeding in the digestive tract [15]. Meanwhile, endoscopic ultrasound (EUS) is a new diagnosis and treatment technology combining gastroscopy and ultrasound. Its principle is to place the micro high-frequency ultrasound probe on the top of the gastroscope. When the gastroscope enters the human body, the situation in the digestive tract can be directly observed through the gastroscope, including changes in tissue, surface morphology, and blood vessels, and images of surrounding tissues and blood vessel structures can be obtained through scanning using the ultrasonic probe at the top of the gastroscope [16–18]. EUS brings convenience to the diagnosis and treatment of PU and GIB, so that clinicians can analyze the gastric lesions of patients through EUS imaging and give timely treatment [19].

Clear imaging is helpful for clinicians to diagnose and treat diseases. In recent years, with the continuous improvement and development of the artificial intelligence algorithm, it has been widely used in image processing in the medical field [20, 21]. Sparse representation theory is a hot topic in the field of image denoising, mainly concerning sparse decomposition and reconstruction algorithm and dictionary design. However, whether images can be sparsely represented is determined by dictionary selection [22, 23]. For dictionary selection, there are usually two methods: one is to select a fixed analysis dictionary, but the sparse representation of samples has limitations, which cannot guarantee the optimal sparse representation of samples; the other is to train and learn according to the existing sample data so as to obtain the supercomplete dictionary library, such as MOD, K-SVD, and joint base dictionary [24]. The study focused on the application value of improved *K*-means Singular Value Decomposition- (N-KSVD-) based ultrasonic image combined with gastroscopy in the diagnosis and analysis of GIB caused by HP.

Accurate diagnosis and timely treatment are very necessary for patients with GIB caused by HP, and a dictionary learning algorithm has good noise reduction effect in ultrasound image combined with gastroscopy. In this study, patients with PU which is highly correlated with HP were selected as the research subjects, and a diagnostic model of N-KSVD-based ultrasonic image combined with gastroscopy was proposed and compared with Discrete Cosine Transform (DCT) algorithm and Global matching dictionary (Global), to evaluate its value in the diagnosis and analysis of GIB caused by HP.

## 2. Materials and Methods

### 2.1. Research Subjects and Grouping

In this study, 86 patients with PU and GIB admitted to our Hospital from June 2018 to June 2020 were selected and defined as the test group and 86 PU patients free of GIB during the same period were selected as the control group. In total, there were 124 males and 48 females. The test group was further divided into HP-positives (60) and HP-negatives (26). This experimental study was approved and supported by the Medical Ethics Committee of the hospital. All participants signed the informed consent form and voluntarily participated in this experiment.

The following are the inclusion criteria: (test group) patients with GIB symptoms such as hematemesis, blood stool, and positive stool occult blood test results; those who did not take any drugs to protect stomach or to affect the test results of HP within 1 week before admission; those who did not take steroid anti-inflammatory drugs within 1 month; and those without major cardiovascular and cerebrovascular diseases. The following are the exclusion criteria: those with the gastric cancer, history of major gastrectomy, and decompensated liver cirrhosis; those with abnormal coagulation function; and those with incomplete clinical data; those with contraindications to ultrasound and gastroscopy examinations.

### 2.2. Ultrasonic Image Combined with Gastroscopy

The patient had the general anesthesia by a professional, and airless distilled water was slowly injected into the stomach cavity while the air in the stomach cavity was drained. Ultrasound endoscopy equipped with miniature high-frequency ultrasound probe was placed 3 cm away from the lesion, and then, a wide range of scanning was carried out from the protrusion of gastric mucosa to lymph nodes around the lesion, and the lesion tissue was collected for biopsy. The frequency of the ultrasound probe (probe frequency: 5~20 MHz) was adjusted according to the specific state of the patient, and the endoscopic ultrasound images of the lesions at different frequencies were obtained. Then, the scanned endoscopic ultrasound image was analyzed for the pathological morphology, surrounding tissue, and echo of ultrasonic signal.

The quantitative analysis software of angiography image was used for image analysis. The analysis data included the relative peak intensity, the rise time (RT), time-to-peak (TTP), and mean transit time (mTT), and the maximum peak intensity of normal stomach tissue was defined as 100%.

### 2.3. Detection of HP

The diagnostic criteria were as per the HP diagnosis standards formulated by the 2nd National Helicobacter Pylori Workshop [25]. Fasting venous blood was drawn from each patient to obtain 1 mL of EDTA anticoagulant. In strict accordance with the operating instructions, a colloidal gold method was used to detect patients with HP IgG antibody (MP biomedical Asia Pacific private Co., Ltd.), and the red infection was positive.

### 2.4. An Ultrasonic Gastroscopy Diagnosis Model Based on N-KSVD

Singular Value Decomposition (SVD) of matrix is an algorithm that diagonalizes the matrix. When applied to image processing, this algorithm can decompose and reconstruct the signal to extract the target signal, so as to achieve noise removal. The K-SVD algorithm is improved on the basis of the *K*-means clustering algorithm. Through SVD decomposition, the largest feature vector is taken as the class center, and K atoms are linearly combined to recover the original signal. The algorithm is divided into two steps: namely, the sparse coding and dictionary update. The mathematical the formula of the sparse model for the K-SVD algorithm is as follows:

(1) m^=arg minmmi0,

where 1 ≤ ‖*n*_*i*_ − *Sm*_*i*_‖ ≤ *ωI* ≤ *W*, and

(2) m^=arg minmni−Smi22+βmi0.

*n*_*i*_ is the untreated sample image, *S* is the training dictionary, and *α* is the *α* maximum tolerance error value. The basic principle of K-SVD algorithm is as follows: under a set of base, the approximate sparse representation *n*_*i*_ of the original signal *m* is obtained and *n*_*i*_ contains good recovery information as much as possible (m^). According to equation (2), through iterations, when the dictionary *S* remains unchanged, the OMP orthogonal matching tracking algorithm is used to find the sparse representation of *N*. After the sparse coding is completed, the dictionary *S* is updated next, and a better dictionary *S* is obtained according to the sparse coefficient matrix *E*.

When the dictionary is updated, the sparse matrix *E* is obtained by sparse coding first. Then, the *t*th column *f*_*t*_ of the dictionary is updated. If the *t*th line corresponding to *f*_*t*_ in the sparse coefficient matrix *E* is expressed as *m*^*t*^_*G*_, the following equation is satisfied:

(3) $$\begin{array}{c} {\left\|N-Sm_{i}\right\|}_{D}^{2}={\left\|N-\overset{t}{\underset{r=t}{\sum }}s_{r}m_{G}^{r}\right\|}^{2}={\left\|\left(N-\overset{t}{\underset{r=t}{\sum }}s_{r}m_{G}^{r}\right)-s_{t}m_{G}^{t}\right\|}^{2}={\left\|H_{t}-s_{t}m_{G}^{t}\right\|}^{2}. \end{array}$$

Then, the algorithm framework of N-KSVD is shown in Figure 1.

### 2.5. Observation Indicators

The following are the grades of blood loss: (i) mild bleeding—blood loss within 0-500 mL, no change in blood pressure, normal heart rate, no change in hemoglobin, and shock index of 0.5; (ii) moderate bleeding—blood loss of 500-1000 mL, decreased blood pressure, heart rate more than 100 beats per minute, hemoglobin 70-100 g/L, accompanied by syncope, oliguria, and thirst, and a shock index of 1.0; and (iii) severe bleeding—blood loss greater than 1500 mL, systolic blood pressure < 80 mmHg, heart rate greater than 120 beats per minute, hemoglobin < 70 g, cold limbs, oliguria, blurred consciousness, and shock index > 1.5, as shown in Figure 2.

The image quality is evaluated factoring into Peak Signal to Noise Ratio (PSNR), Root Mean Square Error (RMSE), and Structural Similarity Index Measurement (SSIM).

Root Mean Square Error (RMSE) is a method to measure the mean error and can evaluate the change degree of data. If s^q,r is the target image, *s* (*q*, *r*)*is* the *original* image, *X* is the horizontal axis pixel of the image, and *Y* is the vertical axis pixel, it is calculated as follows:

(4) $$\begin{array}{c} \text{RMSE}=\frac{1}{X\times Y}\overset{X}{\underset{q=1}{\sum }}\overset{Y}{\underset{r=1}{\sum }}{\left(\overset{\wedge }{s}\left(q,r\right)-s\left(q,r\right)\right)}^{2}. \end{array}$$

The PSNR describes the amount of noise in the image after denoising. Therefore, a higher PSNR value indicates less image noise and better denoising effects.

(5) $$\begin{array}{c} \text{PSNR}=10\log_{10}\frac{255^{2}}{MSE}. \end{array}$$

Image similarity is mainly used to compare the SSIM of the content between two images, and a larger SSIM value indicates better image quality. If *m* and *n* represent the original image and the image to be evaluated, respectively, the mean values *α*_*m*_, *α*_*n*_ represent the image brightness, *ρ*_*m*_, *ρ*_*n*_ represent the image contrast, and *ρ*_*mn*_ represents the image structure. It is calculated as follows:

(6) $$\begin{array}{c} \text{ssim}\left(m,n\right)=\frac{\left(2\alpha_{m}\alpha_{n}+G_{1}\right)\left(2\rho_{mn}+G_{2}\right)}{\left(\alpha_{m}^{2}+\alpha_{n}^{2}+G_{1}\right)\left(\rho_{m}^{2}+\rho_{n}^{2}+G_{2}\right)}. \end{array}$$

### 2.6. Statistical Analysis

The SPSS2.0 is used for the data statistics and analysis on the experimental data. The experimental data are expressed in the mean ± standard deviation ($\bar{x}\pm s$). For measurement data conforming to the normal distribution and *f* test, a *t* test is used for comparison between two samples, *χ*^2^ test is used for the comparison of the classification data, and *I*^2^ is employed to assess the size of the heterogeneity. *P* < 0.05 indicates significant differences among groups.

## 3. Results

### 3.1. Relationship between RMSE and Iteration Times

The experiment explored the relationship between the RMSE and the number of iterations during the dictionary learning based N-KSVD, and the RMSE was recorded when the number of iterations was 1, 10, 20, and 30, as shown in Figure 3. During the training, under 1 cycle of dictionary learning, when the number of iterations was 1, 10, 20, and 30, the RMSE was 11.367, 10.009, 9.7914, and 9.6531, respectively; under 2 cycles of dictionary learning, when the number of iterations was 1, 10, 20, and 30, the RMSE was 11.362, 9.9543, 9.7222, and 9.5889, respectively; under 3 cycles of dictionary learning, when the number of iterations was 1, 10, 20, and 30, the RMSE was 11.352, 9.9395, 9.7025, and 9.549, respectively, and there was no significant difference among them (*P* > 0.05). The test results were similar to those during training.

### 3.2. Denoising Effects of the Three Algorithms

In this experiment, DCT dictionary [26] and Global dictionary [27] were introduced to compare with the N-KSVD algorithm, and the denoising effects of the three algorithms were explored when the noise *ρ* was 10, 30, 50, and 70, respectively, as shown in Figure 4. For the N-KSVD algorithm, when the *ρ* was 10, 30, 50, and 70, the PSNR values after denoising were 35.55, 30.47, 27.91, and 26.08, respectively, and the SSIM values were 0.91, 0.827, 0.763, and 0.709, respectively. It was noted that the PSNR and SSIM values of N-KSVD dictionary after denoising were higher than those of DCT dictionary and Global dictionary, and the difference between N-KSVD dictionary and DCT dictionary was significant (*P* < 0.05).  Figure 5 shows the visual effects of the denoised image processed by the three algorithms. It was noted that the denoising effects based on the N-KSVD dictionary algorithm were the best among the three.

### 3.3. Comparison of Basic Information of Patients

The average age of patients in the test group was 42.68 ± 13.5 years, including 30 females and 56 males; the average age of patients in the control group was 43.45 ± 12.4 years, including 18 females and 68 males. There was no significant difference between the two groups (*P* > 0.05), as shown in Figure 6(a). In the test group, there were 60 HP-positives and 26 HP-negatives, and the difference between the HP-positives and HP-negatives was statistically significant in number (*P* < 0.05), but there was no significant difference in gender and age (*P* > 0.05), as shown in Figure 6(b). The study also compared the positive and negative rates of HP test between the test group and the control group. The results showed that the positive rate in the test group was 69.98% and the positive rate in the control group was 53.25%, with statistical significance (*P* < 0.05).

### 3.4. The Blood Loss, Abdominal Pain, and HP Test Results in the Test Group

Blood loss and abdominal pain of HP-positives and HP-negatives were compared, as shown in Figure 7. As shown in Figure 7(a), mild, moderate, and severe blood loss accounted for 37.66%, 50.02%, and 12.32% of HP-positives in the test group, respectively; for HP-negatives, the corresponding numbers were 32.12%, 48.44%, and 19.44%, respectively, and there was no statistical significance between them (*P* > 0.05). As shown in Figure 7(b), abdominal pain and abdominal tenderness of HP-positives and HP-negatives were compared in the test group. Abdominal tenderness occurred in 39.04% of HP-positives and 38.16% of HP-negatives, respectively, with no significant difference between them; abdominal pain occurred in 59.02% of HP-positives and 37.67% of HP-negatives, respectively, indicating that the number of patients with abdominal pain was higher in HP-positive patients and the difference was statistically significant compared with HP-negative patients (*P* < 0.05).

### 3.5. Imaging Results

For the HP-positives in the test group, 13.8% of patients had ulcers located in the stomach, 74.6% in the duodenum, and 11.6% in the compound condition. For the HP-negatives in the test group, patients with ulcers in the stomach accounted for 17.6%, patients with ulcers in the duodenum accounted for 72.5%, and patients with combined conditions accounted for 9.9%, and the difference was not significant between the HP-positives and HP-negatives in the test group. Then, the size of ulcer was compared. In the test group, HP-positive patients with the diameter between 0 and 1 cm accounted for 71.57%, significantly higher than HP-negatives; HP-positives with the diameter ≥ 1 cm accounted for 28.43%, significantly lower than that of the HP-negatives, and the difference was statistically significant (*P* < 0.05) (Figure 8).

### 3.6. Imaging Data of some Patients

In Case 1, the ultrasonography of a 61-year-old male with gastric ulcer showed a curved stomach (Figure 9(a)).

In Case 2, the ultrasonography of a 52-year-old female with gastric ulcer presented discoid depression on the surface of the large bay of gastric antrum (Figure 9(b)).

## 4. Discussion

PU often occurs in the vicinity of the esophagus, stomach, duodenum, and gastrojejunum anastomosis, but gastric and duodenal ulcers are more common in clinical practice [28]. HP is an important cause of gastric ulcer and duodenal ulcer, and long-term HP colonization will lead to GIB [29].

In this study, a diagnostic model of N-KSVD-based ultrasound combined with gastroscopy was proposed, and DCT dictionary and Global dictionary were introduced for comparative analysis. Then, the relationship between RMSE and the number of iterations during dictionary learning based on N-KSVD was studied, and the RMSE values when the number of iterations was 1, 10, 20, and 30 were compared. The results showed that the updating cycle of N-KSVD dictionary during the iteration process can improve the training and testing performance without many computations. The processing effects of the three algorithms were compared when the noise *ρ* was 10, 30, 50, and 70, respectively. The results showed that the PSNR and SSIM values of N-KSVD dictionary after denoising were both greater than those of DCT dictionary, and the differences were statistically significant, which indicated that N-KSVD dictionary had the best denoising effect, in line with the research results of Grossi et al. [30]. Subsequently, N-KSVD dictionary was used in the diagnosis of patients, and the test group and the control group were compared for basic information. The results showed that the difference between the HP-positive and HP-negative rates was statistically significant (*P* < 0.05), but the difference in gender and age was not significant, consistent with the research results of Cardil et al. [31]. The proportion of HP-positives in the test group was higher than that in the control group, and the difference was significant. Tarhane et al. [32] evaluated 195 patients complaining of abdominal pain, and histopathological examination results showed that 83.58% of them tested positive for HP. Further, HP-positives and HP-negatives were compared for the blood loss and abdominal pain, and it was found that more HP-positives had abdominal pain compared with HP-negatives, and the difference was statistically significant (*P* < 0.05). Finally, the imaging data of patients in the test group were compared, and it was found that patients with duodenal lesions accounted for more than 70% of HP positive and negative patients. The results showed that 71.57% of HP-positives had ulcers with the diameter of 0~1 cm, which was significantly higher than that of HP-negative patients, 28.43% of HP-positives had ulcers with the diameter ≥ 1 cm, which was significantly lower than that in HP-negative patients, and the difference was statistically significant (*P* < 0.05).

## 5. Conclusion

In this study, a diagnostic model of ultrasound combined with gastroscopy based on N-KSVD was proposed, and the DCT dictionary and Global dictionary were introduced for a comparative analysis. The PSNR, RMSD, and SSIM of the three algorithms are compared and analyzed, and the noise reduction performance of N-KSVD dictionary was verified. 86 patients with PU and GIB were selected and defined as the test group, and 86 PU patients free of GIB during the same period were selected as the control group. The results showed that N-KSVD algorithm had a stable performance and a certain noise reduction effect. Ultrasound combined with gastroscopy had an obvious effect on the diagnosis and analysis of HP and GIB. However, some limitations in the study should be noted. The sample size is small, which will reduce the power of the study. In the follow-up, an expanded sample size is necessary to strengthen the findings of the study. In conclusion, this study provides good data support for clinical diagnosis and analysis of HP-induced GIB, for the use of artificial intelligence technology to assist in the diagnosis and treatment of clinical diseases.

## Figures and Tables

**Figure 1:** The framework of the N-KSVD algorithm.

**Figure 2:** The bleeding volume.

**Figure 3:** Relationship between RMSE and the iterative times ((a) during the training and (b) during the test; A: 1 iteration; B: 10 iterations; C: 20 iterations; D: 30 iterations).

**Figure 4:** Noise reduction effects of the three algorithms ((a) noise *ρ* =10; (b) noise *ρ* = 30; (c) noise *ρ* = 50; (d) noise *ρ* = 70). Note: ∗ represents a statistically significant difference compared with N-KSVD (*P* < 0.05).

**Figure 5:** Visual effects of the noise reduction by the three algorithms ((a) the original image; (b) the image with noise; (c) image processed by the DCT dictionary; (d) image processed by the Global dictionary; (e) image processed by the N-KSVD dictionary).

**Figure 6:** Comparison of the basic information of the subjects ((a) shows the age and gender difference between the experimental group and the control group; (b) shows the age and gender differences of HP positive and HP negative in the test group; (c) shows the HP positive and negative rates between the experimental group and the control group). Note: ∗ indicates statistically significant differences compared with HP-negative; # represents a statistically significant difference compared with the test group (*P* < 0.05).

**Figure 7:** The blood loss, abdominal pain, and HP test results in experimental group ((a) shows the amount of blood loss; (b) showed abdominal pain). Note: ∗ represents a statistically significant difference compared with HP negative (*P* < 0.05).

**Figure 8:** Correlation between ulcer location and maximum diameter and HP test results in the test group.

**Figure 9:** Image data of the subjects ((a) case 1; (b) case 2; 1: ultrasonic image, 2: gastroscopic image).

## Data Availability

The data used to support the findings of this study are available from the corresponding author upon request.
